# Histological Changes in Renal, Hepatic and Cardiac Tissues of Wistar Rats after 6 Weeks Treatment with Bipyridine Gold (III) Complex with Dithiocarbamate Ligands

**DOI:** 10.3390/pharmaceutics13101530

**Published:** 2021-09-23

**Authors:** Ahmed Badar, Ayesha Ahmed, Dalal M. Al-Tamimi, Anvarhusein A. Isab, Muhammad Altaf, Sania Ahmed

**Affiliations:** 1 Department of Physiology, College of Medicine, Imam Abdulrahman Bin Faisal University, Dammam 31441, Saudi Arabia; 2 Department of Pathology, College of Medicine, Imam Abdulrahman Bin Faisal University, Dammam 31441, Saudi Arabia; aahmed@iau.edu.sa (A.A.); dtamimi@iau.edu.sa (D.M.A.-T.); 3 Department of Chemistry, King Fahd University of Petroleum and Minerals, Dhahran 31261, Saudi Arabia; aisab@kfupm.edu.sa; 4 Department of Chemistry, Government College University, Lahore 54000, Pakistan; Muhammad.altaf@gcu.edu.pk; 5 Army Medical College, Abid Majeed Road, Rawalpindi 46000, Pakistan; saniaahmed95@hotmail.com

**Keywords:** gold-III compound, bipyridine gold (III)-dithiocarbamate, subacute toxicity, cardiotoxicity, nephrotoxicity, hepatotoxicity

## Abstract

Bipyridine gold (III) dithiocarbamate compounds are Gold-III complexes with promising cytotoxic properties. In this study, the subacute toxicity of a Gold (III) complex with dithiocarbamate ligand was evaluated. In the acute toxicity component, an initial LD_50_ (38.46 mg/kg) was calculated by the administration of 50, 100, 200, 400, and 800 mg/kg of the compound to five groups of rats, respectively (*n* = 4 each). The sixth group was the control. The sub-acute toxicity component comprised the control group A (*n* = 6) and the study groups B (*n* = 10) and C (*n* = 4), which were administered 1 mL distilled water, 1/10 LD_50_ (3.8 mg/kg), and 1/5 LD_50_ (7.6 mg/kg), respectively, daily for 6 weeks. The alive animals were then sacrificed. Autopsy; preservation of renal, hepatic and cardiac tissue in buffered formalin; histopathological processing; microscopic evaluation; and comparison with the controls were sequentially conducted. In the subacute toxicity study at dosages of 3.8 mg/kg and 7.6 mg/kg, the renal tubules remained unaffected with no necrosis or vacuolization. Mild to moderate renal interstitial, hepatic capsular, lobular and portal inflammation along with mild focal hepatic vacuolization were present. At 3.8 mg/kg, the cardiac muscle fibers were unremarkable in 80% (*n* = 8) of the specimens, with mild focal hyalinization in 20% (*n* = 2) of the specimens. The same was observed in 50% (*n* = 2) of the specimens at 7.6 mg/kg. Variable congestion was evident in all of the groups. In the subacute toxicity study, the absence of renal tubular necrosis or vacuolization, the presence of mild inflammatory hepatic and renal alterations, and predominantly unremarkable cardiac muscle fibers suggest that Bipyridine gold (III)-dithiocarbamate is safe in animal studies and is a potential candidate for clinical trials.

## 1. Introduction

The utilization of metal-based compounds for treating cancer started when cisplatin (cis-dichlorodiammine platinum-II) was accidently discovered in the mid-1960s. A long era of development and the utilization of platinum-based drugs started with this discovery. These drugs had very strong anticancerous potential and proved to have a high merit as effective treatment modalities. Their use, however, was hampered by associated tumor resistance and side effects such as nephrotoxicity, hepatotoxicity, neurotoxicity, ototoxicity, myelosuppression, nausea, and dermatological complications [1,2]. This led to research that emphasized formulating and testing alternative metal-based drugs. The present anticancerous medicinal chemistry and drug design aims towards the formulation of novel metal-based organic complexes and compounds with a different pharmacological profile than traditional platinum-based drugs. Due to the effectiveness of cisplatin, the basic concept of developing drugs that are structurally analogous to cisplatin but with different metals was conceived. Structural analogy could preserve anticancer potential in the same way as a platinum compound while the variation in metallic nidus could diminish the platinum-associated adverse side effects.

The medical community has been familiar with the use of gold for a long time. This makes gold complexes readily acceptable. There is evidence that some gold complexes might be useful in cisplatin-resistant tumor cells. Mechanistic studies have reflected that the gold complexes do not interact with DNA as strongly as the platinum complexes do. This points to a different mechanism for cytotoxicity, such as thioredoxin reductase (TrxR) inhibition, COX-1/2 inhibition, DNA damage, cell cycle arrest, ROS accumulation, apoptosis induction, mitochondrial membrane potential changes, angiogenesis inhibition, cellular respiratory inhibition, etc. The proteomic results suggest that gold complexes could affect protein synthesis, energy metabolism, oxidative stress response, and the cytoskeleton. In addition, they may help in the splicing, trafficking, and stability of mRNA [3].

In addition to the antiproliferative properties, the main hinderances to drug development related to gold complexes are stability in the biological media, drug distribution, and target selectivity. This makes complexes with the most suitable ancillary ligands frontrunners. Ligands such as aminophosphines, phosphines, N-heterocyclic carbene, among many others, help transport of the complex in the blood and move across cell membranes to reach the target cells. Some gold complexes such as auranofin are known to have significant antitumor activity and low toxicity. However, some of them produce bioactive metabolites. In fact, this stopped the further development of many gold complexes after initial success [4].

Over the last few years, there have been many studies on the anticancer potential of a number of gold (I) and gold (III) complexes, in particular alkynyl gold derivatives. The water-solubility of phosphine ligands and the good aqueous solution stability of a few heterobimetallic alkynyl gold (I) complexes and trivalent gold (III) alkynyl complexes have made them easy chemicals to work with. Almost all of these studies are in vitro, and despite evidence of encouraging antiproliferative activity and acceptable toxicity profiles, no related complexes have entered clinical trials [5].

With their intrinsic, highly potent tumor anti proliferative potential, gold (III) complexes have recently attained an important role. Their mechanism of action is different from cisplatin [6], but they are electronically and structurally homogenous to platinum (II) compounds [7]. The actual breakthrough for the use of gold compounds will come when these compounds are designed to be more clinically effective and potent, with enhanced cancer cell specificity and selectivity along with diminished organ toxicity [1].

There are limited reports available in the literature that highlight the “in vivo” anticancer potential and cytotoxic characteristics of gold (III) compounds [8,9,10]. Our study group has previously designed and reported on the gold (III) compound [Au(*ethylenediamine*)Cl_2_]Cl and [*trans*-(±)-1,2-(DACH)_2_Au]Cl_3_, where *trans*-(±)-1,2-(DACH) *is Bis(trans-1,2-Diaminocyclohexane)*, which has negligible renal and hepatic organ toxicity compared to other clinically prevalent anticancerous drugs [11].

Gold (III)-dithiocarbamate compounds are a new addition to this evolving series of gold III complexes with new additives. These also have strong anticancer potential, which is inherent to gold III metal containing compounds. These have shown promising anticancer properties involving a different mechanism of action than cisplatin both “in vivo” and “in vitro” [12]. However, studies regarding its organ toxicity are very limited.

In the “in vitro” component of this study, eight new bipyridine gold (III) dithiocarbamate-containing complexes (Figure 1) were synthesized and characterized [13]. These were analyzed and tested in a set of cancer stem cell lines in “in vitro” studies. Compounds 1, 2, 4, 5, 7, and 8 (Figure 1) were seen to have maximum cytotoxicity in Hodgkin lymphoma cells and in ovary, breast, and prostate cancer cell lines. The minimum inhibitory concentration (IC_50_) was seen to be lower than the reference drug cisplatin. Compound 1 (Figure 1 and Figure 2) was observed to be the most active compound in the cisplatin resistant cancer stem lines of ovary and breast cancer, designated as A2780cis and 2780CP-16, respectively [13]. In the current study we evaluated the renal, hepatic, and cardiotoxicity of Compound 1 (bipyridine gold (III) dithiocarbamate-containing complex) in rats who had been administered this compound, with the aim of assessing its vital organ toxicity profile in the context of a new preclinical study for drug development.

## 2. Materials and Methods

This study was conducted at the College of Medicine, Imam Abdulrahman bin Faisal University (IAU), Dammam, Saudi Arabia, in collaboration with the King Fahd University of Petroleum and Minerals (KFUPM), Dhahran, Saudi Arabia (No: IN171005, dated 15 April 2018). The study was conducted following the OECD (Organization for Economic Co-operation and Development) principles of good laboratory practice [14] and was approved by the Institutional Review Board of Imam Abdulrahman Bin Faisal University (formerly the University of Dammam), Saudi Arabia. The acute as well as subacute toxicity study was conducted on Albino Wistar rats obtained from the animal house of IAU. We ensured the use of the minimal number of animals and euthanasia at predetermined end points to minimize the suffering of the animals.

An equal number of male and female rats (*n* = 50), weighing between 200–300 g, were obtained from animal house of Prince Muhammad Research center at Imam Abdulrahman University. The animals were kept in individual cages with standardized room temperature and humidity with free access to food and water for 7 days before the experiment.

### 2.1. Syntheis of Complex (***1***)

The complex (1) [Au(BPY)(DMTC)]Cl_2_(1) was synthesized by stepwise synthesis (Figure 2). Na[AuCl_4_]·2H_2_O, 0.5 mM (200 mg) and 2,2′-Bipyridine 0.5 mM (78 mg) were added simultaneously in 20 mL of ethanol, and the mixture was stirred for 3 h at room temperature. The sodium dimethyldithiocarbamate dihydrate 0.5 mM (72 mg) in 10 mL distilled water was added slowly in the pale-yellow turbid solution obtained from the first step. The reaction mixture was stirred for an additional 1 h at room temperature. The final product appeared as a light-yellow precipitate in the solution. The precipitate was collected by filtration, washed with fresh distilled water (3 × 10 mL), and dried at room temperature under vacuum. Yield: 83.09% (219.98 mg). FT-IR (KBr, υ_max_, cm^−1^): 3570 (m), 3045 (w), 2926 (w); 1586 (m), 1482 (s), 1242 (m), 1159 (w), 1039 (m), 993 (m), 967 (w), 761 (s), 565 (m), 439 (m). ^1^H NMR (500 MHz, DMSO-*d*_6_): δ = 3.36 (6H, 2 × CH_3_), 7.55, 8.06, 8.44, and 8.73 (2H, 2 × CH, BPY). ^13^C NMR (125.1 MHz, DMSO-*d*_6_): δ = 40.29 (CH_3_), 121.65, 125.19, 139.20 and 148.50 (2,2′-BPY), 189.87 (NC = S). Anal. calc. for C_13_H_14_Cl_2_N_3_S_2_Au (544.27): C, 28.69; H, 2.59; N, 7.72; S, 11.78%. Found: C, 28.55; H, 2.51; N, 7.75; S, 11.80%.

### 2.2. Acute Toxicity Study (Single Dose)

In the first step, an approximate LD_50_ was determined by the so called *“staircase method”,* using a small number of animals (two for each dose), testing one dose of the compound-1 bipyridine gold (III) complex with dithiocarbamate ligand at a time (end point at 24 h) and subsequently increasing the dose for the next group if needed. The arbitrarily administered doses of the bipyridine gold (III) complex with dithiocarbamate ligand were 250, 500, and 1000 mg/kg. None of the animals died at 250 mg/kg, one animal became very sick at 500 mg/kg after 20 h and had to be sacrificed, while both of the animals died at 1000 mg/kg: one at 18 h and the other at 22 h. The dose was not increased further. The findings observed in the tissues of the animals used for dose selection are not included with the results of this study.

The five doses where there was the highest change of finding intraperitoneal LD_50_ were then chosen a. These were 50, 100, 200, 400, and 800 mg/kg. These doses were then given to five groups of rats, with four animals in each group. A sixth group with four animals served as the control and was injected with distilled water. The animals were kept under continuous observation for the initial 2 h and were then sequentially observed every 2 h for any symptoms of toxicity to avoid the rodents experiencing any suffering. At the end of 24 h, the number of rats that had died in each group were counted. The percentage of animals that had died at each dose level were transformed to probits [15], and LD_50_ was then determined according to the method of Miller and Tainter [16]. All of the living animals were sacrificed and dissected at the end of the 24 h period. The kidneys, livers as well as hearts of the animals were collected and preserved in 10% formalin for histological examination. The LD_50_ determined by the probits was 38.46 mg/kg body weight (Table 1).

### 2.3. Subacute Toxicity Study

A total of 20 rats of same age and approximately same weight (200–250 g) were used for this arm of the study, which continued for 42 days. Each rat was housed in a separate cage. The cages were kept at standardized temperature and humidity for one week before the start of intervention. They were given free access to food (rat-chow) and water. Food consumption was assessed daily by evaluating the leftover food, whereas the body weight of each rat was determined once before the commencement of treatment and weekly thereafter at a fixed time of the day.

Group-A (the control group, *n* = 6) was injected with 1 mL of distilled water daily for 6 weeks by intraperitoneal injection. Group-B (*n* = 10) was injected 1/10 of LD_50,_ a dose of 3.8 mg/kg body weight, daily for 6 weeks by intraperitoneal injection. Group-C (*n* = 4) was injected 1/5 of LD_50_ for 7.6 mg/kg bodyweight daily for 6 weeks by intraperitoneal injection. The day of death was noted for the animals that died during the 6 weeks, and tissues were removed by dissection. At the end of 6 weeks, the alive animals were sacrificed. Tissues of all of the animals were put in 10% formaldehyde and were sent for histological evaluation (Table 2).

### 2.4. Histopathological Evaluation

An automated tissue processor (Tissue–tek VIP-5, from SAKURA) was employed for tissue processing. An initial two step fixation consisting of two cycles of two hours each for tissue immersion in buffered formalin was followed by washing the tissue in distilled water for half an hour for the removal of the fixative. The tissue was dehydrated by exposing it to an increasing concentration of alcohol, i.e., 70%, 90%, and 100% for variable time periods, followed by clearing by the sequential immersion of the tissue in a mixture 50% xylene and alcohol and then pure xylene for half an hour each. The tissue was then impregnated in molten wax followed by embedding, formation of paraffin blocks, thin sectioning at 4–5 um thickness, and, finally, hematoxylin and eosin (H&E) staining. The prepared slides were then evaluated for histopathological alterations [17].

H&E-stained sections of renal, hepatic, and cardiac tissue from the rats administered the gold III compound and the control rats were examined for tubulopathies including necrosis, apoptosis, and tubular vacuolization. Additional findings of inflammation and vascular changes such as congestion were also noted in the renal tissue. Renal tubular necrosis was graded as follows: [18]

Grade 0 = unremarkable renal tubules.

Grade 1 = renal tubular epithelial cell degeneration without significant apoptosis or necrosis.

Grades 2–5 = renal tubular epithelial cell degeneration including apoptosis and necrosis comprising <25%, <50%, <75%, and ≥75% of the renal tubules.

The hepatic tissue was evaluated for alterations in the architecture, portal triads, hepatocytes, sinusoids, inflammation, and the presence of degeneration, necrosis, and fatty change. These alterations were grouped into one of the following categories: [19]

Hepatitis: Acute, chronic, cholestatic, granulomatous.

Steatosis, steatohepatitis: microvesicular or macrovesicular.

Cholestasis: Bland or chlolestatic hepatitis.

Vascular Abnormalities: sinusoidal obstruction syndrome.

The cardiac tissue was analyzed for cytoplasmic vacuolization, variation in cardiac muscle fiber size, the hyalinization of muscle cells, fibrosis, muscle necrosis with contraction band formation, altered staining properties, and myocytolysis. Interstitial inflammation and interstitial edema were also noted. The extent of the changes was semi-quantitatively graded as follows: [20,21]

Grade 0: Unremarkable histological findings (0%).

Grade 1: Mild change involving up to a 30%; initiation of change.

Grade 2: Moderate change involving 31–60%.

Grade 3: Severe change involving 61–100%; widespread changes identified.

### 2.5. Analysis

The results are summarized as frequencies arranged as crosstabs and were compared for significance using the chi square test in SPSS-IBM version 21.

## 3. Results

### 3.1. Acute Toxicity Study

In acute toxicity study in Group 1, with a dose of 50 mg/kg, two out of four animals died before being euthanized for autopsy. In Group 2, 4, and 5, with dosages of 100, 400, and 800 mg/kg, respectively, all of the animals died before being euthanized, and Group 3, with a dose of 200 mg/kg, in which three animals had died. Additionally, all the animals in these respective groups showed signs of increased motor activity, either before death or before being euthanized. Group 6 was the control group, which all of the animals remained alive. The following tables and figures show the renal (Table 3 and Table 4, Figure 3 and Figure 4), hepatic (Table 5 and Table 6, Figure 5 and Figure 6), and cardiac (Table 7 and Figure 6) microscopic findings.

### 3.2. Sub-Acute Toxicity Study

This phase was divided into three groups. The first, Group A, which had six animals, was the control group. The renal, hepatic, and cardiac tissue were all unremarkable, as shown in Table 8 and Figure 7.

The second group, “B”. had 10 animals who were given a dosage of **3.8 mg/kg (1/10 of LD50)** body weight (dosage planned for 6 weeks). However, two of the animals, B1 and B2, died on day 22 and 32, respectively. (Table 8).

The third group, “C”, had four animals who were given a dosage of **7.6 mg/kg (1/5 of LD50)** body weight (dosage planned for 6 weeks). However, C1 and C2 were sacrificed on day 37, and C3 and C4 died on day 35 and 36, respectively (Table 8).

None of the animals in Group B or C had any signs of acute toxicity. However, two animals, C1 and C2, were sacrificed when signs of distress started to appear.

The histological findings are presented in Table 8 and Figure 8.

## 4. Discussion

Nephrotoxicity with concomitant renal failure is a major drawback in platinum-based anticancer drugs, especially cisplatin. This can present as acute tubular injury manifesting histologically as renal tubular cellular necrosis with inflammation. The process of necrosis can involve several necrosis inducing pathways that may include mitochondrial permeability transition-induced regulated necrosis, necroptosis, ferroptosis, or parthanatos [22]. Cisplatin, the major anti-cancerous agent in solid tumors, has nephrotoxity as its major initial and long-term drawback that can also lead to drug resistance. Its renal accumulation and concentration with reduced renal perfusion manifests morphologically as necrosis of the proximal tubular terminal portion and apoptosis, mainly the distal nephron [23]. In our bipyridine gold (III) complex with dicarbamato ligand, there was no evidence of renal tubular necrosis in either of the doses used in our subacute toxicity study (Figure 8 and Table 8).

In subacute toxicity with a dose of 3.8 mg/kg or 7.6 mg/kg, the renal tubules remained unaffected, with no evidence of necrosis or renal tubular vacuolization. Mild to moderate congestion was seen. At a dose of 3.8 mg/kg, mild to moderate focal interstitial inflammation was seen in three specimens (30%). A dose of 7.6 mg/kg produced mild to moderate interstitial inflammation in two (50%) of the study animals l (Figure 8 and Table 8). This finding suggests that the bipyridine gold (III) complex with dicarbamato ligand compound is safe renal wise.

As previously reported, the complex has proven its merit as a potent anticancer compound. This compound ligand was shown to have a low IC_50_ value, a high cellular uptake, and showed highly potent cytotoxicity against prostatic, ovarian, breast, lung, and Hodgkin lymphoma cells. It was proven to be 60–80-fold more active than cisplatin in inhibiting cellular proliferation in cisplatin resistant cells comprising a clone A2780cis of ovarian adenocarcinoma and s MCF-7 clone of breast cancer cells [13]. Therefore, a high anticancerous potency specifically against cisplatin resistant cancer stem lines and preserved renal tubules merits this complex to be investigated further in the context of new drug development.

Oxiplatin, a third-generation platinum compound used in many malignancies, is less nephrotoxic compared to other platinum-based drugs. However, it has also been reported to induce renal tubular acidosis and/or necrosis. Oxaliplatin is a substrate for both the organic cation transporters (OCT2) present in proximal tubular basolateral membranes and the multidrug and toxin extrusion transport proteins (MATE, especially MATE2) present in proximal tubular brush border. An imbalance between OCT and MATE caused by platinum-based drugs lead to its diminished renal extrusion. Platinum compounds hence accumulate in renal tubules with concomitant renal damage [24]. It could be postulated that in the sub-acute toxicity study, the levels of MATE could be decreased by our bipyridine Gold (III) dicarbamato complex, which leads to its renal expulsion and hence preserved renal histology.

In the acute toxicity part of our study, however, grade 1 necrosis was seen. (Figure 3 and Table 3) The bipyridine gold (III) dicarbamato complex in the previously reported part of the study was proven to be a pro-apoptotic compound, and its anticancerous activity is exerted by inhibiting cellular proliferation by enhancing the mitochondrial intrinsic apoptotic pathway by a time-dependent activation of caspase 3 and 9, the promotion of mitochondrial permeability, and the release of cytochrome-c. All of these lead to the induction of apoptosis, evidenced by the fragmentation of the DNA analyzed by Apo-Direct analysis [13]. As such, the induction of apoptosis or grade 1 renal tubular necrosis seen in the acute toxicity part of the study could have been caused by the renal accumulation of the compound with this mechanism of action.

Renal tubular vacuolization was seen in the acute toxicity study (Figure 3 and Table 3). It has rarely been reported. Oxaplatin-induced renal tubular vacuolization was reported by Jobayari et al. [24]. It has also been reported after the administration of many types of drugs such as cisplatin, cyclophosphamide, immunoglobulins, sirolimus, imatinib, desferasirox, and cyclosporine [25], and hyperosmotic fluids, such as inulin, glucose, mannitol, sucrose, and radiocontrast agent, etc. [26]. Again, renal drug accumulation is considered to be the plausible mechanism. These findings and possible mechanisms imply that the bipyridine gold (III) dicarbamate complex that is under study accumulated in the renal tubules to cause minimal renal tubular necrosis and vacuolization. In sub-acute toxicity, however, the levels of the accumulated drug were so minimal that no renal damage occurred at histological levels (Figure 8 and Table 8). Such observations need to be validated by further investigations at the molecular level.

Another finding seen in the acute toxicity (Figure 4 and Table 4) and sub-acute toxicity parts (Figure 8 and Table 8) of the study is plasmacytic pyelitis and interstitial inflammation. Drugs can lead to an immunological reaction or a hapten-mediated disease, leading to renal damage. Drugs can act as an antigen with immune complex formation, leading to development of acute glomerulonephritis or acute interstitial nephritis. In the hapten mediated disease, part of a drug, any metabolite of the drug, or any substance modified by the drug can act as a hapten. These haptens can bind to the tubular epithelium or interstitial matrix, eliciting an immune reaction. This immune reaction can be an allergic reaction with involvement of IgE and eosinophils or it could be a cell-mediated immune reaction conducted by CD4+ T lymphocytes [27]. These drug-related immune reactions are categorized as idiosyncratic or Type B reactions. These are unrelated to the mechanism of action of the drug [22]. The production of inflammasomes by the drug can also be considered as a possible mechanism that induces interstitial inflammation [28]. Cisplatin may also activate complex signaling pathways, including inflammatory pathways [29]. The extent of inflammation seen in sub-acute toxicity with our compound was predominantly mild and focal. This level of inflammatory changes needs to be evaluated clinically, and blood tests need to be conducted to assess the extent of renal impairment; however, in the absence of other findings of renal damage such as necrosis and tubular vacuolization, these seem to be of relatively less significance.

Regarding the hepatic tissue, in the sub-acute toxicity study at a dose of 3.8 mg/kg and 7.6 mg/kg, the hepatic tissue only showed inflammatory changes comprising mild capsular acute inflammation, mild to moderate focal lobular and portal inflammation, and, occasionally, mild focal cytoplasmic vacuolization (Figure 8 and Table 8). In acute toxicity part of the study, the toxic effects were more apparent, with appearance of mild steatosis in all groups and a graded pattern of individual cellular degeneration/necrosis as well as increased cytoplasmic vacuolization along with inflammatory changes (Figure 5 and Table 5). Congestion was a finding that was seen to varying extents the in acute, sub-acute, and control groups.

The liver is the main organ involved in drug metabolism and clearance and is therefore the most susceptible to drug induced liver injury. This mode of hepatic injury is the main reason for the termination of drugs in clinical trials and the withdrawal of drugs used for treatment purposes. This may have a dose dependent or an idiosyncratic dose independent presentation [30].

Massive hepatotoxicity is seen with cisplatin, doxorubicin, and 5- Flurouracil (5-FU), even at therapeutic doses. In a study by El-Sayyad et al., treatment at low doses of 0.2 mg/kg body weight of cisplatin and doxorubicin or 10 mg/kg of 5-FU in rats for 20 days was shown to induce hepatic cellular vacuolar degeneration and apoptosis along with vascular alterations comprising endothelial cell damage with perivascular mononuclear cellular infiltration and periportal fibrosis. A dose of 1 mg/kg body weight, the therapeutic dose of cisplatin and doxorubicin, led to hepatocellular necrosis with dissolution of the hepatic cords with dense inflammatory cellular infiltration. An increased tendency for hepatic fibrosis and granulomatous lesions was observed with doxorubicin treatment. Cisplatin and doxorubicin showed more hepatic damage compared to the treatment with 5-FU [31].

Mild capsular inflammation, mild lobular and portal inflammation, and mild congestion are the findings that were seen in the sub-acute toxicity part of the study, (Figure 8 and Table 8); however, the same changes were observed in the controls (Figure 7 and Table 8). The presence of these findings in low-dose and drug-free animals implies that some other mechanism was responsible for these alterations. The drug-induced mechanism is not the only plausible mechanism that can cause these inflammatory changes.

Regarding steatosis, drug-induced steatosis or steatohepatitis is reported in less than 2% of cases of nonalcoholic steatohepatitis (NASH). Drugs that can induce NASH may show a definite metabolic alteration, such as tamoxifen, which involves the decreased incorporation of free fatty acids into very low-density lipoproteins along with their decreased hepatic expulsion or can be independent of any known definite mechanism, such as perhexiline maleate or amiodarone, or may produce sporadic cases of NASH, such as carbamazepine [32,33]. In the conversion of hepatocytes of acetyl-CoA to fatty acids is regulated by sterol regulatory element-binding protein-1c, a membrane-bound transcription factor that can activate fatty acid synthase, acetyl-CoA carboxylase, stearoyl-CoA desaturase, and ATP-citrate lyase, leading to lipogenesis. Lipid hemostasis is also modulated by another transcription factor, the peroxisome proliferator-activated receptors. The mitochondrial accumulation of drugs with resultant interference in mitochondrial electron transport chain and β-oxidation can also cause drug-induced liver injury and NASH [34,35]. The basic mechanism that underlies the development of steatosis in our compound has yet to be unraveled, but it can safely be stated that the lack of steatosis in the sub-acute toxicity study renders this compound as a hepatic-safe compound. However, such observations need to be validated with more extensive clinical and biochemical studies.

Hepatocytic individual cell degeneration/necrosis was seen in the acute toxicity study (Figure 5 and Table 5). Drug-induced hepatocytic necrosis may include massive, sub massive, and zonal necrosis. The combined pattern of necrosis and inflammation seen in drug-induced liver injury may include massive, sub massive, and zonal necrosis. Massive necrosis is characterized by pan-acinar necrosis with the complete loss of hepatocytes and parenchymal collapse between the residual portal areas. It has been shown to involve multiple contiguous acini. Ductular proliferation, varying extents of portal inflammation, and evidence of regeneration in the remaining hepatic parenchyma is also seen. Necrosis involving zone 3 is a feature of zonal necrosis. There is usually no associated portal or parenchymal inflammation. Zonal necrosis is seen to have some chemotherapeutic agents [36]. The necrosis seen with our compound, even in very high doses, was very minimal, and there was no necrosis observed in the sub-acute toxicity study, imparting the attribute of hepatic safety to this compound.

The cardiac findings in the sub-acute toxicity part (Figure 8 and Table 8) with a dosage of 3.8 mg/kg cardiac muscle fibers were unremarkable in 80% (*n* = 8). Mild cardiac muscle fiber hyalinization was seen in 20% (*n* = 2) of specimens in less than 10% of the material examined. Pericardial acute inflammatory cellular infiltrate was seen in 10% (*n* = 1). A dosage of 7.6 mg/kg led to mild focal hyalinized fibers in 50% of specimens (*n* = 2). In the acute toxicity study (Figure 6 and Table 7), the cardiac histological alterations were mild cytoplasmic vacuolization in all specimens, mild to moderate hyalinization, and congestion. Congestion was a finding that was also seen in the controls and in the sub-acute toxicity study.

Cardiac hyalinization and fibrosis manifesting as cardiomyopathy is a side effect of many anti-cancerous agents. Doxorubicin, an effective anticancerous agent that is widely used in the treatment of solid tumors has an associated cardiomyopathy that has been seen histologically as areas of and scattered vacuolated cardiomyocytes and foci of patchy and widespread cardiac interstitial fibrosis. When the acute damage is healed, fibroblastic proliferation with histiocytic infiltration is seen in healed areas [37]. Doxorubicin kills cancerous cells by intercalating into DNA with topoisomerase II (TOP2) inhibition and caspase activation [38]. Its cardiotoxic effects are mainly manifested by the generation of reactive oxygen species [39]. New bipyridine gold (III) dithiocarbamate-containing complexes (the compound in this study) have been previously reported to overproduce mitochondrial reactive oxygen species [13]. Their cardiac hyalinization and vacuolization may be attributed to this mechanism. However, the damage observed in our cases was not that extensive, as only focal cytoplasmic vacuolization and hyalinized fibres were seen in the sub-acute toxicity study (Figure 8 and Table 8).

As far as cytoplasmic vacuolization is concerned, it has been reported to be reversible, transient, or irreversible. Vacuolar formation could just be an adaptation to a variety of environmental alterations [40]. Its transient form is mostly caused by weak basic amine-containing lipophilic compounds that can pass through cell and organellar membranes, increasing intraorganellar osmotic pressure with water diffusion and the development of vacuolization. Irreversible vacuolization results due to cytotoxic stimulus with cytopathological damage culminate as cell death [41]. This pattern of vacuolization may be caused by caspase-independent cell death mechanisms comprising oncosis, methuosis, necroptosis, or paraptosis [42]. We had vacuolization in cardiac specimens in the acute and sub-acute toxicity parts of the study. Whether this was just an adaptive response or an initiation of cell death needs to be elaborated upon with more studies at molecular levels. The changes observed, however, seem to be adaptive and reversible, as no evidence of necrosis was discerned in cardiac tissue, even at high doses in the acute toxicity part of the study.

Drug resistance to chemotherapeutic agents is a central problem in oncology. The results of this investigation have identified a new class of gold (III) compounds as potential candidates for application in cancer chemotherapy. This is based on the demonstration that gold (III) compounds are effective in cisplatin-resistant cell lines. Moreover, since these compounds contain a dithiocarbamate group that is capable of preventing a reaction with other sulfur-containing proteins, we hypothesize a reduced toxicity in vivo. Thus, a gold (III) drug with an appropriate ligand, such as that presented in this study, has the potential to be an alternative to platinum-based drugs in cancer treatment.

Conclusion: In the subacute toxicity part of the study with a dose of 3.8 mg/kg or 7.6 mg/kg, the renal tubules remained unaffected, with no evidence of necrosis or renal tubular vacuolization. The cardiac muscle fibers also remained unremarkable in 80% of the specimens, with mild focal muscle fiber hyalinization seen in the remaining 20%. Mild focal renal and hepatic inflammatory changes were the only concomitant alterations. Such minimal histological alterations may attribute this bipyridine gold (III) complex with dithiocarbamates ligand to be safe in animal studies and strongly suggest it as a potential candidate for clinical trials.

## Figures and Tables

**Figure 1:** The bipyridine gold (III) dithiocarbamate-containing complexes **(1–8)**.

**Figure 2:** The synthesis of Complex (**1**).

**Figure 3:** Renal tubular histological alterations as seen in acute toxicity study. (**a**): Renal tubular necrosis grade 1, H&E, ×20. (**b**): Renal tubular necrosis grade 1. Individual cell apoptosis can also be seen. H&E, ×40. (**c**): Renal tubular cytoplasmic vacuolization H&E, ×40. (**d**): Renal tubular cytoplasmic vacuolization with an occasional individual cell apoptosis, H&E, ×40.

**Figure 4:** Spectrum of renal inflammatory changes as seen in acute toxicity study. (**a**): Moderate renal interstitial inflammation, H&E, ×20. (**b**): Moderate renal interstitial inflammation, H&E, ×40. (**c**): moderate plasmacytic pyelitis, H&E, ×20. (**d**): moderate plasmacytic pyelitis, H&E, ×40.

**Figure 5:** Hepatic histological alterations as seen in acute toxicity study. (**a**): Mixed hepatic micro and macrovesicular steatosis. An occasional apoptotic hepatocyte is also seen, H&E, ×40. (**b**): Mixed hepatic micro and macrovesicular steatosis, H&E, ×40. (**c**): Mild acute capsular inflammation, H&E, ×40. (**d**): Mild cytoplasmic vacuolization, H&E, ×40.

**Figure 6:** Cardiac histological findings as seen in acute toxicity study. (**a**): Moderate cardiac muscle fiber hyalinization, H&E, ×20. (**b**): Moderate cardiac muscle fiber hyalinization, H&E, ×40. (**c**): Marked cardiac congestion, H&E, ×20. (**d**): Mild cardiac cytoplasmic vacuolization, H&E, ×40.

**Figure 7:** Unremarkable renal (**a**), hepatic (**b**), and cardiac (**c**) tissue, as seen in controls of sub-acute toxicity, H&E, and ×20.

**Figure 8:** Histological picture of renal hepatic and cardiac tissue in subacute toxicity study at a dose of 3.8 mg/kg. (**a**): Unremarkable renal tissue as seen in sub-acute toxicity (3.8 mg/kg), H&E, ×40. (**b**): Mild renal interstitial inflammation as seen in sub-acute toxicity (3.8 mg/kg), H&E, ×40. (**c**): Unremarkable hepatic tissue as seen in sub-acute toxicity (3.8 mg/kg), H&E, ×40. (**d**): Mild hepatic cytoplasmic vacuolization as seen in sub-acute toxicity (3.8 mg/kg), H&E, ×40. (**e**): Unremarkable cardiac tissue as seen in sub-acute toxicity (3.8 mg/kg), H&E, ×40. (**f**): Mild focal cardiac hyalinization and congestion as seen in sub-acute toxicity (3.8 mg/kg), H&E, ×40.

**Table 1:** Determination of the lethal doses of gold complex for the determination of LD50 after intraperitoneal injection in rats (*n* = 24, 4 in each group).

Group	Dose (mg/kg)	Log Dose	% Dead	Probits
1	50	3.912	50	0.585
2	100	4.605	100	0.783
3	200	5.298	75	0.912
4	400	5.991	100	0.973
5	800	6.685	100	0.994
Control	0	0	0	0

**Table 2:** Disposal of animals in subacute study (*n* = 20).

Animal No.	Treatment	Fate (Upto 42 Days)
A1–A6	Distilled water	All survived, sacrificed on day 42, tissues preserved for histopathology
B3	3.8 mg/kg BW (1/10 of LD_50_)	Died on day 22, tissues preserved for histopathology
B9		Died on day 32, tissues preserved for histopathology
B1, B2, B4–B8, B10		Survived up to day 42, sacrificed, tissues preserved for histopathology
C1	7.6 mg/kg BW (1/5 of LD_50_)	Sacrificed on day 37 due to animal distress, tissues preserved for histopathology
C2		Sacrificed on day 37 due to animal distress, tissues preserved for histopathology
C3		Died on day 35, tissues preserved for histopathology
C4		Died on day 36, tissues preserved for histopathology

**Table 3:** Renal tubular necrosis and vacuolization in acute toxicity study. (*n* = 24).

Groups (*n* = 4 in Each Group)	Dose mg/kg	Renal Tubular Necrosis Grade						Renal Tubular Vacuolization		
		5	4	3	2	1	0	None	Less Than 50%	More Than 50%
**1**	50	0	0	0	0	25% (*n* = 1) **Figure 3a,b**	75% ^#^ (*n* = 3)	100% ^#^ (*n* = 4)	0	0
**2**	100	0	0	0	0	50% (*n* = 2)	50% (*n* = 2)	75% ^#^ (*n* = 3)	25% (*n* = 1) **Figure 3c,d**	0
**3**	200	0	0	0	0	25% (*n* = 1)	75% ^#^ (*n* = 3)	50% (*n* = 2)	50% (*n* = 2)	0
**4**	400	0	0	0	0	50% (*n* = 2)	50% (*n* = 2)	25% (*n* = 1)	75% ^#^ (*n* = 3)	0
**5**	800	0	0	0	0	25% (*n* = 1))	75% ^#^ (*n* = 3)	25% (*n* = 1)	75% ^#^ (*n* = 3)	0
**6** **(control)**	-	0	0	0	0	0	0	0	0	0

^#^: *p* Value < 0.05 on Χ^2^ test.

**Table 4:** Pyelitis/interstitial inflammation and congestion in renal tissue in acute toxicity study (*n* = 24).

Groups (*n* = 4 in Each Group)	Dose mg/kg	Pyelitis/Interstitial Inflammation %			Congestion %		
		None	Mild	Mod/ Marked	None	Mild	Mod/ Marked
**1**	50	75% ^#^ (*n* = 3)	25% (*n* = 1)	0	0	50% (*n* = 2)	50% (*n* = 2)
**2**	100	75% ^#^ (*n* = 3)	25% (*n* = 1)	0	0	0	100% ^#^ (*n* = 4)
**3**	200	0	75% ^#^ (*n* = 3)	25% (*n* = 1) **Figure 4a–d**	0	25% (*n* = 1)	75% ^#^ (*n* = 3)
**4**	400	25% (*n* = 1)	25% (*n* = 1)	50% (*n* = 2)	0	0	100% ^#^ (*n* = 4)
**5**	800	0	25% (*n* = 1)	75% ^#^ (*n* = 3)	0	25% (*n* = 1)	75% ^#^ (*n* = 3)
**6** **(control)**	-	0	0	0	0	0	0

^#^: *p* Value < 0.05 on Χ^2^ test.

**Table 5:** Extent of hepatic steatosis, necrosis, and congestion in acute toxicity study (*n* = 24).

Groups (*n* = 4 in Each Group	Dose mg/kg	Steatosis			Hepatocellular Necrosis/Degeneration			Congestion		
		None	Mild	Moderate Marked	None	Individual Cell Degeneration	Necrosis with Inflammation	None	Mild	Mod/ Marked
**1**	50	75% ^#^ (*n* = 3)	25% (*n* = 1) **Figure 5a,b**	0	100% ^#^ (*n* = 4)	0	0	0	75% ^#^ (*n* = 3)	25% (*n* = 1)
**2**	100	75% ^#^ (*n* = 3)	25% (*n* = 1)	0	75% ^#^ (*n* = 3)	25% (*n* = 1)	0	25% (*n* = 1)	75% ^#^ (*n* = 3))	0
**3**	200	75% ^#^ (*n* = 3)	25% (*n* = 1)	0	100% ^#^ (*n* = 4)	0	0	0	50% (*n* = 2)	50% (*n* = 2)
**4**	400	75% ^#^ (*n* = 3)	25% (*n* = 1)	0	25% (*n* = 1)	75% ^#^ (*n* = 3)	0	0	0	100% ^#^ (*n* = 4)
**5**	800	0	100% ^#^ (*n* = 4)	0	0	100% ^#^ (*n* = 4)	0	0	25% (*n* = 1)	75 ^#^ (*n* = 3)
**6 (control)**	-	100% ^#^ (*n* = 4)	0	0	100% ^#^ (*n* = 4)	0	0	25% (*n* = 1)	75 ^#^ (*n* = 3)	0

^#^: *p* Value < 0.05 on Χ^2^ test.

**Table 6:** Extent of portal, lobular, and capsular inflammation and cytoplasmic vacuolization in hepatic tissue in acute toxicity study (*n* = 24).

Groups (*n* = 4 in Each Group)	Dose mg/kg	Inflammation Portal/Lobular			Capsular Acute Inflammation			Cytoplasmic Vacuolization		
		None	Mild	Moderate/ Marked	None	Mild	Mod/ Marked	None	Mild	Moderate/ Marked
**1**	50	75% ^#^ (*n* = 3)	25% (*n* = 1)	0	25% (*n* = 1)	75% ^#^ (*n* = 3) **Figure 5c**	0	25% (*n* = 1)	75% ^#^ (*n* = 3) **Figure 5d**	0
**2**	100	50% (*n* = 2)	50% (*n* = 2)	0	50% (*n* = 2)	50% (*n* = 2)	0	25% (*n* = 1)	75% ^#^ (*n* = 3)	0
**3**	200	75% ^#^ (*n* = 3)	25% (*n* = 1)	0	50% (*n* = 2)	25% (*n* = 1)	25% (*n* = 1)	0	50% (*n* = 2)	50% (*n* = 2)
**4**	400	25% (*n* = 1)	75% ^#^ (*n* = 3)	0	0	100% ^#^ (*n* = 4)	0	0	75% ^#^ (*n* = 3)	25% (*n* = 1)
**5**	800	0	100% (*n* = 4)	0	50% (*n* = 2)	50% (*n* = 2)	0	0	75% ^#^ (*n* = 3)	25% (*n* = 1)
**6 (control)**	-	75% ^#^ (*n* = 3)	25% (*n* = 1)	0	50% (*n* = 2)	50% (*n* = 2)	0	75% (*n* = 3)	25% (*n* = 1)	0

^#^: *p* Value < 0.05 on Χ^2^ test.

**Table 7:** Cardiac histological findings in acute toxicity study (*n* = 24).

Groups (*n* = 4 in Each Group)	Dose mg/kg	Cytoplasmic Vacuolization				Hyalinization				Congestion		
		None	Mild	Mod	Marked	None	Mild	Mod	Marked	None	Mild	Mod/ marked
**1**	50	75% ^#^ (*n* = 3)	25% (*n* = 1)	0	0	75% ^#^ (*n* = 3)	25% (*n* = 1)	0	0	0	50% (*n* = 2)	50% (*n* = 2))
**2**	100	25% (*n* = 1)	75% ^#^ (*n* = 3)	0	0	25% (*n* = 1)	75% ^#^ (*n* = 3)	25% (*n* = 1) **Figure 6a,b**	0	0	0	100% ^#^ (*n* = 4)
**3**	200	50% (*n* = 2)	50% (*n* = 2))	0	0		75% ^#^ (*n* = 3)	0	0	0	50% (*n* = 2)	50% (*n* = 2) **Figure 6c**
**4**	400	75% ^#^ (*n* = 3)	25% (*n* = 1)	0	0	75% ^#^ (*n* = 3)	25% (*n* = 1)	75 (*n* = 3)	0	0	0	100% ^#^ (*n* = 4)
**5**	800	50% (*n* = 2)	50% **Figure 6d**	0	0		100% ^#^ (*n* = 4)	0	0	0	25% (*n* = 1)	75% ^#^ (*n* = 3)
**6** **(control)**	-	0	0	0	0	0	0	0	0	25% (*n* = 1)	75% ^#^ (*n* = 3)	0

^#^: *p* Value < 0.05 on Χ^2^ test.

**Table 8:** Histological findings in sub-acute toxicity study with of the doses of 3.8 mg/kg and 7.6 mg/kg (*n* = 20).

Animal Groups	Dose	RENAL				HEPATIC					CARDIAC	
		Normal	Necrosis	Interstitial Inflammation		Normal	Portal/Lobular Inflammation		Mild Capsular Inflammation ***	Mild Cytoplasmic Vacuolization ***	Normal	Mild Focal Cardiac Fiber Hyalinization <10% of Tissue Examined
				Mild	Mod		Mild	Mod				
**A Control** **(*n* = 6)**	**0**	**100%** **#** **(*n* = 6)** **Figure 7a**	**0**	**0**	**0**	**67% ^#^** **(*n* = 4)** **Figure 7b**	**33%** **(*n* = 2)**	0	16% (*n* = 1)	0	100% ^#^ (*n* = 6) **Figure 7c**	0
B * (*n* = 10)	3.8 mg/kg	70% ^#^ (*n* = 7)	0	20% (*n* = 2) **Figure 8a,b**	10% (*n* = 1)	70% ^#^ (*n* = 7)	20% (*n* = 2)	10% (*n* = 1)	20% (*n* = 2)	10% (*n* = 1) **Figure 8c,d**	80% ^#^ (*n* = 8)	20% (*n* = 2) **Figure 8e,f**
C ** (*n* = 4)	7.6 mg/kg	50% ^#^ (*n* = 2)	0	25% (*n* = 1)	25% (*n* = 1)	50% (*n* = 2)	50% (*n* = 2)	0	0	50% (*n* = 2)	50% (*n* = 2)	50% (*n* = 2)

^#^: *p* Value < 0.05 on Χ^2^ test. * One specimen showing pericardial acute inflammatory infiltrate was seen in B. ** Mild plasmacytic pyelitis was also seen in C4 in renal tissue. *** Mild capsular inflammation and cytoplasmic vacuolization was seen in the same animals as those showing portal and lobular inflammation. Varying extents of congestion were seen in all groups, including the control group.

## Data Availability

Not applicable.
